# Key Proteins of Activating Cell Death Can Be Predicted through a Kainic Acid-Induced Excitotoxic Stress

**DOI:** 10.1155/2015/478975

**Published:** 2015-01-28

**Authors:** Hsiu-Ling Tsai, Sue-Joan Chang

**Affiliations:** ^1^Department of Food Nutrition, Chung Hwa University of Medical Technology, Jente, No. 89, Wunhua 1st Street, Rende District, Tainan City 717, Taiwan; ^2^Department of Life Sciences, National Cheng Kung University, Tainan 701, Taiwan

## Abstract

Epilepsy is a major neurological disorder characterized by spontaneous seizures accompanied by neurophysiological changes. Repeated seizures can damage the brain as neuronal death occurs. A better understanding of the mechanisms of brain cell death could facilitate the discovery of novel treatments for neurological disorders such as epilepsy. In this study, a model of kainic acid- (KA-) induced neuronal death was established to investigate the early protein markers associated with apoptotic cell death due to excitotoxic damage in the rat cortex. The results indicated that KA induces both apoptotic and necrotic cell death in the cortex. Incubation with high concentrations (5 and 500 *μ*M, >75%) and low concentrations (0.5 pM: 95% and 50 nM: 8%) of KA for 180 min led to necrotic and apoptotic cell death, respectively. Moreover, proteomic analysis using two-dimensional gel electrophoresis and mass spectrometry demonstrated that antiapoptotic proteins, including heat shock protein 70, 3-mercaptopyruvate sulfurtransferase, tubulin-B-5, and pyruvate dehydrogenase E1 component subunit beta, were significantly higher in apoptosis than in necrosis induced by KA. Our findings provide direct evidence that several proteins are associated with apoptotic and necrotic cell death in excitotoxicity model. The results indicate that these proteins can be apoptotic biomarkers from the early stages of cell death.

## 1. Introduction

Epilepsy is a major neurological disorder characterized by spontaneous seizures (discharges) accompanied by motor and/or perceptual dysfunction. Recently, researchers have proposed that the underlying pathological mechanisms of epilepsy are excessive activation of excitatory amino acid (EAA) receptors, with accompanying generation of reactive oxygen species (ROS) [1, 2]. Studies have demonstrated the relationship between oxidative stress and epileptic seizures in animal models, with markedly increased mitochondrial superoxide production and intracellular Ca^2+^ concentration ([Ca^2+^]_i_) [3], or mitochondrial dysfunction [4]. A growing number of* in vivo* and* in vitro* studies have also confirmed that oxidative stress induces cell death in excitotoxic injury [5, 6].

Several experimental models of epileptic seizures have been developed using EAA receptor agonists such as lithium-pilocarpine or kainic acid (KA). KA is an agonist of the *α*-amino-3-hydroxy-5-methyl-4-isoxazolepropionic acid (AMPA) subtype of EAA receptors and is widely used to study the mechanisms behind neurological disorders by creating models of cell damage. KA has been reported to induce excitotoxic cell death in immature and adult animals by systemic or intraventricular injection and in primary cultures and* in vitro* neuronal cell lines [7, 8]. Two types of neuronal death, including apoptosis and necrosis, have been proposed to occur in the KA models. A number of studies have reported that apoptosis was the major mode of cell death, while a few studies have suggested the existence of KA-induced necrotic cell death, as well as the coexistence of apoptosis and necrosis in the brain [9, 10].

Apoptosis and necrosis are two main types of cell death both with distinct morphological and molecular features. Apoptosis is described as an active, well-regulated, and energy-dependent form of cell death. In contrast, necrosis represents a passive, less orderly, non-energy-requiring form. In the past two decades many studies have reported the toxic events ultimately leading to cell death through disturbed homeostasis, such as excess ROS production [11], ATP-generation blocking [12], or activation of death receptors (such as the Fas/CD95/Apo1 receptor [13], TNF receptor [14], or the NMDA receptor [15]). The main proteins involved in determining the mode of cell death, be it by apoptosis or necrosis, remain unclear. The present study aimed to provide direct evidence for the involvement of different proteins in the two modes of neuronal death. The study was designed to identify and compare protein expression patterns in apoptosis and necrosis of cortical cells through an excitotoxicity-induced neuronal cell death model.

## 2. Materials and Methods

### 2.1. Isolation of Dissociated Immature Cortical Cells

Dissociated immature cortical cells from 14-day-old Sprague-Dawley rats (purchased from the Animal Center of the Medical College, National Cheng Kung University, Tainan, Taiwan) were prepared by collagenase A (0.33 mg/mL) digestion at 37°C for 30 min in a shaking bath. After washing with Eagle's minimal essential medium (MEM, GIBCO), the cells were cultured in MEM with 10% fetal bovine serum and maintained for 24 h at 37°C in an atmosphere of 95% air and 5% CO_2_. The density of the dissociated immature cortical cells (mixed neuronal and glial cells) was adjusted to 10^6^ cells/mL for KA induction.

### 2.2. Kainic Acid (KA) Induction

KA (Sigma) was prepared as a concentrated stock solution (1 mM) in the cell culture medium. Dissociated immature cortical cells were treated with KA at the concentrations of 0.005 pM to 500 *μ*M (0.005 pM, 0.5 pM, 50 nM, 5 *μ*M, and 500 *μ*M) for 5, 30, 60, and 180 min at 37°C in a shaking water bath, under an atmosphere of 95% O_2_/5% CO_2_. Each concentration and duration of application was analyzed in triplicate. The methods used to characterize the cellular responses of cortical cells to excitotoxic insults induced by KA are described below.

### 2.3. Flow Cytometric Measurement of Intracellular Oxidative Stress in Immature Cortical Cells after KA Induction

Flow cytometric analysis was undertaken to investigate KA excitatory neurotoxicity and its relationship to quantitative changes in ROS, [Ca^2+^]_i_, and mitochondrial membrane potential (MMP). Briefly, 1 mL of dissociated immature cortical cells (10^6^ cells) treated with KA at five different concentrations for four different induction times as mentioned above was incubated with fluorescent dye. ROS generation was measured using 2′,7′-dichlorofluorescein diacetate (DCFH-DA, final concentration 5 *μ*M) [16]. [Ca^2+^]_i_ was detected with a calcium-binding dye Fluo-3 AM [17]. MMP was detected with 3-3′-dihexyloxacarbocyanine (DiOC6) [18]. The mixtures were incubated at 37°C for 30 min in the dark and washed twice with PBS, and the fluorescence intensity of the samples was measured in 5000 dissociated cells with an EPICS XL-MCL flow cytometer (Coulter, Miami, FL, USA) by gating FL1 (emission at 525 nm).

### 2.4. Apoptosis and Necrosis Detection

*(1) Determination of Necrotic Cell Death by Flow Cytometry*. The number of necrotic cells was measured using the method described by Harrison et al. [17]. Briefly, propidium iodide (PI, final concentration 4.5 *μ*g/mL) was added to cells treated with KA (10^6^ cells/mL) and then incubated for 20 min at room temperature in the dark. After washing twice with PBS, the fluorescence intensity of the samples was measured with an EPICS XL-MCL flow cytometer (Coulter) by gating FL3 (emission at 615 nm) using 5000 dissociated cells. The results are expressed as the percentage of cell death compared with vehicle-treated controls.

*(2) Determination of Apoptosis by DNA Fragmentation.* DNA was extracted from the cells using the Blood and Tissue Genomic DNA Mini Kit (Viogene, Taipei, Taiwan). The percentage of DNA fragmentation was analyzed by conventional agarose gel electrophoresis as reported previously [19]. Twenty micrograms of DNA from each sample was electrophoresed on a 1.2% agarose gel containing 0.5% ethidium bromide at a 4 V/cm gel length (30 V for 6 h). The gels, in the presence or absence of DNA “laddering” of approximately 200 base pairs, were then photographed under ultraviolet light.

*(3) Determination of Apoptosis by Annexin V Staining*. The ratio of apoptosis was assessed using Annexin V, as reported previously [20]. Specimens of cortex were diluted to a concentration of 1 × 10^5^ cells/mL with PBS. 20 *μ*L of cell suspension was spread onto a slide and 5 *μ*L FITC-Annexin V and 50 *μ*L Annexin-binding buffer (BD Biosciences) were added. After staining for 15 min at room temperature in the dark, the slides were observed under a fluorescence microscope (Axioskop; Zeiss, Germany) with an excitation filter of 515–560 nm and a barrier filter of 590 nm. Images were captured using the Komet 3.1 image analysis system (Kinetic Imaging, Bromborough, UK).

### 2.5. Preparation of Sample for Two-Dimensional Gel Electrophoresis (2-DE)

After the occurrence of apoptosis was confirmed by these tests, two KA-treated samples (0.5 and 5 *μ*M KA-induced excitotoxic insult for 3 h) were added to a 1 mL lysis buffer containing 7 M urea, 2 M thiourea, 4% 3-[(3-cholamidopropyl) dimethylammonio]-1-propanesulfonate (Chaps), 40 mM Tris, and 10 mM dithiothreitol plus phosphatase/protease inhibitors (1 mM Na_3_VO_4_, 1 mM PMSF) on ice and shaken for 30 minutes to extract the proteins. The supernatant was purified using the Amersham 2D clean-up kit (GE Healthcare Biosciences, Australia) and the protein pellet was finally resuspended in a 250 *μ*L rehydration buffer (8 M urea, 2% w/v CHAPS, 15 mM DTT, and 0.5% v/v IPG buffer, pH 3–10). Total protein was determined using the Micro BCA Protein Assay reagent and bovine serum albumin as a standard.

Two-dimensional electrophoresis (2-DE) was performed as described previously [21]. The first dimension, isoelectric focusing (IEF), was performed using 18 cm immobilized pH gradient (IPG) gel strips (pH 4–7). This dimension separates proteins in the mixture based on their isoelectric points (PI) following a stepwise incremental voltage program: 30 V for 16 h, 500 V for 1 h, 1 KV for 1 h, and 8 KV for 4 h, with a total power of 34 kV-h. The second dimension was performed using 11% SDS polyacrylamide gels (Protean II xi cell, Bio-Rad, CA, USA) at 40 mA/gel for 1 h. The gels were then fixed in 40% ethanol and 10% acetic acid in water overnight and stained with 0.25% w/v silver nitrate solution containing 0.02% formaldehyde for 30 min.

### 2.6. 2-DE Data Analysis

The stained 2-DE gels were scanned using ImageScanner operated by LABSCAN 3.01 software (Amersham Biosciences). Image analysis was carried out using the software IMAGEMASTER 2D (version 2002.1, Amersham Biosciences). Each spot intensity volume was processed using background subtraction and total spot volume normalization, which produced the spot volume percentage (% vol.). Each cell sample (0.5 and 5 *μ*M KA-induced excitotoxic insult for 3 h) was subjected to 2-DE three times to minimize run-to-run variation. A reference gel was artificially created and used to match corresponding protein spots between gels. Spot intensities (spot volume) were then normalized as a percentage of the total spot volume using spots that were present in all gels (% vol.). Spots with a % vol. ratio between the two groups of greater than 1.5 were regarded as dysregulated and were selected for subsequent destaining (50% acetonitrile and 25 mM ammonium bicarbonate). These samples were digested overnight at 37°C (10 *μ*L of 0.1 *μ*g/*μ*L of trypsin digestion buffer in 25 mM ammonium bicarbonate). After centrifuging at 2000 ×g for 10 min, the supernatant was subjected to mass spectrometry analysis for protein identification. The in-gel digestion, mass spectrometry analysis, and database search were commissioned by the Departments of Environmental and Occupational Health, National Cheng Kung University College of Medicine, Taiwan.

### 2.7. Statistical Analysis

Flow cytometry data were analyzed by analysis of variance using SAS statistical software (SAS Institute, Inc.). Data from the different groups were compared using the one-way ANOVA method followed by Duncan's test (*P* < 0.01).

## 3. Results

### 3.1. ROS Changes in Dissociated Immature Cortical Cells Treated with KA

KA exhibited an excitotoxic effect by generating significant amounts of ROS in dissociated immature cortical cells at five different concentrations (ranging from 0.005 pM to 500 *μ*M) and over four different time periods (5, 30, 60, and 180 min), as shown in Figures 1(a)–1(e). Compared to the untreated controls at the same time, the application of moderate and high doses of KA (0.5 pM, 50 nM, 5 *μ*M, and 500 *μ*M) resulted in significantly higher ROS production. No significant change was detected in ROS generation at the lowest dose of KA (0.005 pM) (*P* < 0.01 versus control). Compared to the group treated with a moderate dose of KA (0.5 pM) group, ROS generation was markedly increased at 30, 60, and 180 min in the group treated with high concentrations of KA (5 and 500 *μ*M) (*P* < 0.01 versus 0.5 pM KA group) (Figure 1(f)). Comparison of ROS production at the same concentration of KA at different time periods showed that KA induced a time-dependent increase in intracellular ROS production.

### 3.2. Changes in MMP in Dissociated Immature Cortical Cells Treated with KA

Figures 2(a)–2(e) illustrate the effects of different doses of KA on excitotoxic changes in MMP at all time points. A significant reduction in MMP (indicated by an increased fluorescent intensity) in dissociated immature cortical cells occurred with all KA concentrations and incubation times compared to cells without KA administration (*P* < 0.01 versus control). Treatment with 50 nM of KA for 60 or 180 min and 5 *μ*M and 500 *μ*M of KA for 5, 30, 60, or 180 min caused significant decreases in MMP compared to the moderate dose of KA (0.5 pM; *P* < 0.01 versus 0.5 pM KA group). In this study, there were significant differences in ROS production and decreased MMP in all KA groups.

### 3.3. Changes in Intracellular [Ca^2+^] in Dissociated Immature Cortical Cells Treated with KA

KA-induced intracellular calcium changes and neurotoxicity were observed in cortical cells; however, there was no consistent KA concentration response (Figures 3(a)–3(e)). High concentrations of KA (5 and 500 *μ*M) applied over 30 min, moderate doses of KA (0.5 pM and 50 nM), and 0.005 pM KA at four time points caused a rapid rise in [Ca^2+^]_i_ compared to untreated cells (*P* < 0.01 versus control). However, the administration of high concentrations of KA (5 or 500 *μ*M) for only 5 min significantly reduced intracellular Ca^2+^ levels (*P* < 0.01). When compared with 0.5 pM KA group over 60 min, there were significant increases in intracellular Ca^2+^ levels at the highest concentrations of KA (5 and 500 *μ*M) and with moderately high concentrations of KA (*P* < 0.01 5, 500 *μ*M and 50 nM KA versus 0.5 pM KA group) (Figure 3(f)). There were large decreases in intracellular Ca^2+^ levels in cells exposed to the highest concentrations of KA (5 and 500 *μ*M) compared to cells exposed to 0.5 pM KA for 5 or 30 min. Prolonged exposure of cultured cortical cells to the same concentration of KA did not produce a time-dependent increase in intracellular calcium ion levels.

### 3.4. Determination of Necrotic Cell Death of Immature Cortical Cells Treated with KA

The excitotoxicity-associated necrotic cell death following KA treatment was quantified using the DNA fluorescent dye, propidium iodide (PI). Our results showed that KA induced significantly more necrotic cell death (>70% of the neurons) at higher concentrations (5 and 500 *μ*M) applied over 180 min than those in control group (*P* < 0.01; Figure 4). If the same two concentrations of KA (5 and 500 *μ*M) were applied over 30 min, the percentage of necrotic cells increased from approximately 8% to 12%. Therefore, these results indicate that necrotic cell death is associated with KA and there is a significant exposure-time effect at high KA concentrations. No significant effects of KA on necrotic cell death were found at lower concentrations of KA (0.005 pM, 0.5 pM, and 50 nM), even with incubation periods of 180 min.

### 3.5. Determination of Apoptosis by Annexin V and DNA Fragmentation Assays

KA-induced excitotoxic apoptosis in rat cortical cells was confirmed by both DNA fragmentation and Annexin V. DNA fragmentation is the nuclear hallmark of apoptosis and was found to occur in this study following 3 hr of 0.5 pM KA exposure. Low levels of DNA fragmentation occurred after 50 nM KA exposure. Neither controls nor cells treated with 5 *μ*M KA demonstrated DNA fragmentation (Figure 5). The Annexin V assay produced the same result in cells exposed to 50 nM KA (Figure 6). Using fluorescence microscopy, a high percentage of Annexin V-positive cells (approximately 95%) were observed in the samples treated with 0.5 pM KA for 180 min (Figures 6(a) and 6(b)). Fewer Annexin V-positive cells (approximately 8%) occurred in the samples treated with 50 nM KA for 180 min (Figures 6(c) and 6(d)). There were no Annexin V-positive cells among the control samples (Figures 6(e) and 6(f)). Through the above measures, apoptosis was found to be induced at moderate concentrations of KA (0.5 pM and 50 nM) and necrosis at high concentrations (5 *μ*M) in rat cortical cells.

### 3.6. Candidate Proteins Associated with Apoptosis versus Necrosis under Excitotoxic Conditions

The protein spots that differed between the apoptotic and necrotic groups were subjected to mass spectrometry for protein identification. Five 2-DE protein spots revealed significant differences between the two groups (Figure 7).  Table 1 provides a summary of four proteins, heat shock protein 70, 3-mercaptopyruvate sulfurtransferase, tubulin *β*-5, and pyruvate dehydrogenase E1 component subunit beta, which were significantly upregulated (1.5-fold or greater) in cells that had undergone apoptotic death. There were no significant differences in the intensities of guanine nucleotide binding protein (<1.5-fold) between the apoptosis and necrosis groups. Mass spectrometry was unable to identify the remaining three spots (data not shown), indicating that there were no MS/MS data matching with the sequences from a mass spectra database search. Mass spectrometry of these proteins and the probability based Mowse scores obtained with the Mascot search engine are shown in Figure 8.

## 4. Discussion

In our previous study, we used pilocarpine, another cholinergic neurotoxin, to induce experimental models of status epilepticus and found that pilocarpine induced two types of seizures: severe prolonged seizures and repeated seizures [22]. The findings of the study indicated that the animals in the group with prolonged seizures had excessive levels of reactive oxygen species and malondialdehyde production and lower activities of superoxide dismutase and catalase as compared with the group with repeated seizures. Therefore, in the current study we aimed to investigate the proteins involved in different types of oxidative damage in the brain. We found that the two modalities of cortical cell death (apoptosis and necrosis) in dissociated immature cortical cells exposed to excitotoxic insults were present by flow cytometry and were confirmed by PI staining, DNA fragmentation, and Annexin V assay. 2-DE gel analysis and mass spectrometry demonstrated differential protein profiles in apoptosis and necrosis, enabling elucidation of the regulated mechanisms of cell death.

ROS are important for the mediation of cell survival and proliferation. However, excessive ROS generation is a well-known major contributing factor to excitatory amino acid neurotoxicity and neurodegenerative diseases resulting from oxidative stress [1, 23]. In this study, quantitative flow cytometry was used to evaluate the extent of oxidative stress in dissociated cortical cells in rats exposed to KA-induced excitotoxicity. An increase in intracellular ROS levels occurred in our* in vitro* KA models of excitotoxicity. An association between excitotoxicity and an increase in ROS has also been demonstrated in previous* in vivo* studies [1, 24]. Large amounts of ROS represent the main cause of cell damage and ultimately promote cell death [25]. Time- and dose-dependent effects of KA on ROS production in cortical cultures are consistent with the findings from previous reports in hippocampal cultures [26]. In cortical cultures, high concentrations of KA (5 and 500 *μ*M) promoted higher levels of ROS production than those found in cells exposed to moderate KA concentrations (0.5 pM). Furthermore, KA also induced a time-dependent increase in intracellular ROS production.

Mitochondria, the site of ATP generation, are thought to be involved in the pathway to cell death through changes to or loss of MMP [4, 27]. The findings of the present study are consistent with previous studies that have demonstrated depolarization of mitochondrial membranes in injured cells in response to activation of metabotropic glutamate receptors [28, 29]. In another study, MMP levels were reduced in cells and cells became less viable after exposure to high concentrations of carbonyl cyanide 3-chlorophenylhydrazone [30]. The type of cell death invoked might depend on the intensity of the stimulus [31]. Increased ROS generation accompanied by mitochondrial damage participates in neuronal cell death.

Since the first reported cell death due to excitotoxic effects in the CNS in 1969, it has been shown that alterations in calcium homeostasis play key roles in excitotoxicity [3, 32]. In this study, an increase in [Ca^2+^]_i_ occurred in cells exposed to KA treatment as compared with untreated cells. However, a decrease in [Ca^2+^]_i_ was also observed in cells exposed to high doses of KA (5 and 500 *μ*M) for 5 minutes. A similar finding was reported by Youn and Randić [33], who discovered that application of KA (3 *μ*M, 2 min) significantly depressed C fiber monosynaptic excitatory postsynaptic potentials through the kainate receptor, GluR5. It is likely that in the present study the varying effects of different doses of KA on [Ca^2+^]_i_ were due to the selection of metabotropic and ionotropic receptor entry into cells. In the CNS, Ca^2+^ influx via receptor-mediated mechanisms reportedly mediates cell death [34]. This in turn results in the activation of a variety of intracellular signals and, ultimately, different neurotoxic effects. One study suggested that excessive Ca^2+^ loading contributes to cell death in some cell types [35]. In this study, excessive Ca^2+^ loading occurred after exposure to a high concentration of KA for over 60 min. Excessive Ca^2+^ loading may therefore contribute to mitochondrial depolarization followed by the opening of permeability transition pores and a concurrent significant increase in ROS levels. Based on the theory that injurious stimuli of a lesser amplitude than those causing necrosis in the same cells induce apoptosis [36], 5 and 500 *μ*M concentrations of KA and a 0.5 pM concentration of KA applied for 3 h may result in different types of oxidative stress.

In this study, high concentrations of KA (5 and 500 *μ*M) caused an increase in the percentage of necrotic cells after 3 hours of exposure, which was confirmed by PI staining. Results obtained by flow cytometry demonstrated the presence of both necrotic and nonnecrotic cells in these samples. A widely accepted biomarker of apoptosis is Annexin V [19]. In the current study, almost 95% of cells underwent KA-induced cell death following exposure to 0.5 pM KA for 3 h and demonstrated apoptotic bodies (fluorescence signals) under light and fluorescence microscopy and Annexin V assay. In contrast, only a few apoptotic cells were observed in cells exposed to 50 nM KA for 3 h, and no apoptotic cells were observed in the control cells. The presence of DNA ladders, or internucleosomal genomic DNA fragmentation, is a biochemical hallmark of apoptosis and was visualized in this study using agarose gel electrophoresis in cells treated for 3 h with 0.5 pM KA. However, the control cells remained dark without any DNA laddering, and no typical ladders of DNA fragments occurred in necrotic cells (5 *μ*M KA for 3 h). From the above results, it can be inferred that KA led to cortical cell death after 3 hours of exposure via either apoptosis or necrosis, depending on the concentration administered. The result is consistent with the finding of an* in vivo* epileptic study showing that the apoptotic component of seizure-induced neuronal death in the high-dose KA group versus the low-dose KA group is insult duration- or severity-dependent [37].

Identification of death-mediating factors through a model of excitotoxicity has the potential to aid the prediction of outcomes and lead to better targeting of interventions and management strategies. Thus, the present study aimed to identify and characterize key proteins involved in apoptotic versus necrotic cell death. 2D gel electrophoresis and mass spectrometry- (MS-) based proteomics were used to analyze KA-induced apoptosis and necrosis by examining differences in protein expression profiles. Proteins spots in which the silver intensity was increased by more than 1.5-fold in KA-induced apoptosis compared with the same protein in necrotic cells under MS spectrometry were selected for analysis. Analyses identified one such spot as tubulin. Tubulin is, reportedly, an antiapoptotic protein involved in the apoptotic morphology. Previous research has suggested that the levels of tubulin mRNA transiently increase during apoptosis and that events occurring downstream from tubulin binding are critical for the generation of apoptosis [38]. Tubulin is also the biochemical target for several anticancer drugs [39]. Pyruvate dehydrogenase E1 component subunit beta, also known as an antiapoptotic protein, was significantly induced in response to excitotoxicity in this study. Its upregulation in KA insult-induced apoptotic death indicated a relative resistance to KA treatment. This response was also observed by Gerner and coworkers [40]. Pyruvate dehydrogenase acts as a bridge between glycolysis and the tricarboxylic acid cycle [41]. Its increase in the present study indicated the activation of the aerobic pathway required for apoptosis, as opposed to pathways involved in necrosis or critical illnesses. These results are consistent with those of Concannon and colleagues [42], who found that AMPK activation and Bim couple transient energy depletion occurred in response to stress-induced neuronal apoptosis in excitotoxicity. Pyruvate dehydrogenase also has a role in other conditions, such as cardiac ischemia and reperfusion injury [43]. Even postischemic hearts show improvement after pharmacological stimulation with pyruvate dehydrogenase [44]. In addition, we observed an increase in the level of a third protein, 3-mercaptopyruvate sulfurtransferase. This is reportedly an antioxidant protein with important roles in the maintenance of redox homeostasis and the production of hydrogen sulfide (H_2_S) in normal tissues including the brain [45]. H_2_S is a synaptic modulator and neuroprotectant and may protect the heart against ischemic injury by a pathway involving protein kinase C [46]. The final protein that exhibited the greatest increase in expression (2.2-fold) in apoptotic cells compared to necrotic cells was heat shock protein 60 (HSP60). HSP70, a cytosolic HSP, plays an antiapoptotic role in excitotoxicity, cerebral ischemia, and myocardial injury and has been intensively investigated. In contrast, mitochondrial matrix HSP60 is more controversial and has been reported to have both antiapoptotic and proapoptotic effects on cells. A proapoptotic role of HSP60 was found in surgical specimens from patients with intractable epilepsy, whereas the antiapoptotic gene Bcl-2 was downregulated to less than 50% of the normal level [47]. Similar to our results, Kirchhoff et al. [48] suggested that overexpression of HSP60 exerted an antiapoptotic effect to increase the survival rate of cardiac myocytes undergoing myocardial injury. These results indicated that the dual role of HSP60 is mediated through its interaction with other heat shock proteins, which suggests that there exist cooperative effects of heat shock proteins in protecting cells from injury and facilitating cell recovery and survival [49]. In our model of KA-induced cortical cell excitotoxicity and apoptosis, these proteins, all of which were antioxidant and antiapoptotic proteins, were significantly activated. The expressions of these proteins suggest the presence of an inducible defense system in apoptotic death that prevents the development of necrosis. Under ER stress conditions, the fate of cells is dependent on the balance between antiapoptotic genes in cell adaptive responses and proapoptotic genes in cell death responses [50]. As a consequence, the balance between the antiapoptotic and proapoptotic effectors or proteins may be critical for determining the cell fate, even in different cell types.

## 5. Conclusion

The functional role of the differentially expressed proteins implies the involvement of apoptosis and not necrosis in excitotoxic brain cortical cell death. Our study demonstrates different protein expression in cells undergoing apoptotic versus necrotic cell death and holds the potential for new treatment strategies for apoptotic death resulting from excitotoxic disease processes. Further research on the complex interactions between these apoptotic proteins as mediators in cell death may validate their role in diseases such as epilepsy.

## Figures and Tables

**Figure 1:** Comparison of intracellular reactive oxygen species (ROS) measured by flow cytometry following exposure to kainic acid (KA) over different time periods. (a–e) Representative fluorescence histograms obtained from dissociated cortical neurons (10^6^ cells/mL) from 14-day-old rat brains incubated with 2′,7′-dichlorofluorescein diacetate in the presence of 0.005 pM, 0.5 pM, 50 nM, 5 *μ*M, and 500 *μ*M KA for 5 (red), 30 (yellow), 60 (blue), and 180 min (purple). The white curve represents the background fluorescence of untreated neurons; the colored curves represent the increased fluorescent intensity of neurons following KA treatment (a shift to the right versus white curve). (f) Bar graphs of ROS levels (mean ± SE) expressed as percentage change in mean fluorescence intensity (MFI) from controls. Experiments were performed in triplicate, and statistical analyses of the data were performed using ANOVA. Data are expressed as percentage change from controls. ^#^ *P* < 0.01 compared with the respective time period in the control group. ^*^ *P* < 0.01 compared with the respective time period in the 0.5 pM KA group. Apoptosis and necrosis labels indicate the degrees of cell death at 180 min of treatment.

**Figure 2:** Comparison of mitochondrial membrane potential (MMP) measured by flow cytometry following exposure to kainic acid (KA) over different time periods. (a–e) Representative fluorescence histograms obtained from dissociated cortical neurons (10^6^ cells/mL) from 14-day-old rat brains incubated with 3-3′-dihexyloxacarbocyanine in the presence of 0.005 pM, 0.5 pM, 50 nM, 5 *μ*M, and 500 *μ*M KA for 5 (red), 30 (yellow), 60 (blue), and 180 min (purple). The white curves represent the background fluorescence of untreated neurons; the colored curves represent the increased loss of MMP from cells (indicated by an increase in 535 nm fluorescence intensity versus white curve) following KA treatment. (f) Bar graphs of MMP intensity (mean ± SE) expressed as the percentage change in mean fluorescence intensity (MFI) from controls. Experiments were performed in triplicate, and statistical analyses of the data were performed using ANOVA. Data are expressed as percentage (%) change from controls. ^#^ *P* < 0.01 compared with the respective time period in the control group. ^*^ *P* < 0.01 compared with the respective time period in the 0.5 pM KA group. Apoptosis and necrosis labels indicate the degrees of cell death at 180 min of treatment.

**Figure 3:** Comparison of intracellular calcium ion concentration ([Ca^2+^]_i_) measured by flow cytometry following exposure to different doses of kainic acid (KA) over different time periods. (a–e) Representative three-dimensional graph obtained from dissociated cortical neurons (10^6^ cells/mL) from 14-day-old rat brains incubated with Fluo-3 AM in the presence of 0.005 pM, 0.5 pM, 50 nM, 5 *μ*M, and 500 *μ*M KA for 5 (red), 30 (yellow), 60 (blue), and 180 min (purple). The white curves represent the background fluorescence of untreated neurons; the colored curves represent the decreased or increased fluorescent intensity of neurons following KA treatment (a shift to the left or right, resp., versus white curve). (f) Bar graphs of intracellular calcium concentration (mean ± SE) expressed as the percentage change in mean fluorescence intensity (MFI) from controls. Experiments were performed in triplicate, and statistical analyses of the data were performed using ANOVA. Data are expressed as percentage change from controls. ^#^ *P* < 0.01 compared with the respective time period in the control group. ^*^ *P* < 0.01 compared with the respective time period in the 0.5 pM KA group. Apoptosis and necrosis labels indicate the degrees of cell death at 180 min of treatment.

**Figure 4:** Effects of kainic acid (KA) on necrotic cell death measured using propidium iodide (PI) staining and flow cytometry of dissociated cortical neurons (10^6^ cells/mL) from 14-day-old rat brains exposed to 0.005 pM to 500 *μ*M KA for 5, 30, 60, or 180 min. Bar graphs show the amount of necrotic cell death (mean ± SE) expressed as the percentage change in mean fluorescence intensity (MFI) from controls. Experiments were performed in triplicate, and statistical analyses of the data were performed using ANOVA. Data are expressed as the percentage change from controls. ^#^ *P* < 0.01 compared with the respective time period in the control group.

**Figure 5:** DNA ladder formation shown by gel electrophoresis. DNA was prepared from dissociated cortical cells from neonatal rats (P14) exposed to 0.5 pM, 50 nM, and 5 *μ*M kainic acid (KA) for 180 min, as well as from a control group. The DNA mixture was separated by 1.5% agarose gel. Lane 1 shows no DNA fragments in the cells from untreated dissociated cortical cells. Lanes 2 and 3 show no DNA fragments in the dissociated cortical cells treated with 5 *μ*M and 50 nM KA for 180 min. Lane 4 shows DNA fragments from dissociated cortical cells treated with 0.5 pM KA for 180 min.

**Figure 6:** Morphology of apoptotic bodies in cells treated with 0.5 pM and 50 nM kainic (KA) acid and control cells. 20 *μ*L of dissociated cortical neurons (1 × 10^5^ cells/mL) exposed to 0.5 pM ((a) and (b)) and 50 nM (c and d) KA for 180 min and control cells ((e) and (f)) were spread onto a slide and 5 *μ*L of FITC-Annexin V and 50 *μ*L Annexin-binding buffer were added. The slides were subsequently analyzed using fluorescence microscopy ((a), (c), and (e)) or light microscopy ((b), (d), and (f)) for the detection of apoptosis. Apoptotic cells (Annexin V-positive, black arrows) were visualized in KA-treated groups ((a) and (c)) under fluorescence microscopy but were not detected in control cells (e). Blue arrows indicate the corresponding Annexin V-positive cells in KA-treated groups as seen under light microscope.

**Figure 7:** Comparison of electrophoretic protein profiles from apoptotic and necrotic cells. Following 180 min of treatment with 0.5 pM and 5 *μ*M kainic acid (KA), each dissociated cortical neuron cell lysate was separated into three different two-dimensional gel electrophoresis (2-DE) runs and stained with silver-stain. Figures are from representative gels demonstrating typical protein profiles of 5 *μ*M induced necrotic cells (a) and 0.5 pM KA-induced apoptotic cells (b). More than 1500 protein spots were routinely detected. The red circles indicate protein spots that were altered significantly by at least 1.5-fold with a resulting increase in apoptotic cells compared with necrotic cells based on data from at least three independent gels (*P* < 0.05).

**Figure 8:** Mascot search results for four significantly upregulated proteins in kainic acid-induced apoptosis based on probability based Mowse scores using the Mascot search engine. Possible proteins matched to the spectral masses with differential Mowse scores are shown as multiple bars on the *x*-axis. Only proteins with Mowse scores greater than 64 (outside the shaded area) were considered statistically significantly different (*P* < 0.05). Proteins (without black arrow) were excluded if their masses corresponded to those for trypsin or keratins or to other irrelevant proteins. Black arrows indicate the Mowse score of 3-mercaptopyruvate sulfurtransferase, pyruvate dehydrogenase beta, tubulin beta 5, and heat shock protein 60 (HSP60).

**Table 1:** Summary of five differentially regulated proteins in kainic acid-induced apoptosis, compared to KA-induced necrosis, as detected by two-dimensional differential in-gel electrophoresis (DIGE) and mass spectrometry.

Spot number	Protein	Accession (ID) number^a^	MW (Da)^b^/PI	Change^c^	Sequence Coverage (%)^d^	Mowse score^e^
1^*^	3-Mercaptopyruvate sulfurtransferase	NP_620198.1	32809/5.88	1.6	13%	67
2^*^	Pyruvate dehydrogenase beta	NP_001007621.1	35842/6.20	1.7	27%	185
3^*^	Tubulin beta 5	NP_035785.1	49639/4.78	1.8	9%	112
4^*^	Heat shock protein 60 (HSP60)	CAA37654.1	57890/5.35	2.2	19%	252
5	Guanine nucleotide binding protein	NP_001013932.1	37339/5.74	1.2	16%	122

^*^Significantly upregulated proteins demonstrated a greater than 1.5-fold increase in expression.

^a^Reference for protein identification from the protein database at the National Center for Biotechnical Information (NCBI).

^b^MW: molecular weight.

^c^Intensity of spots from two samples run in the 2D-DIGE gel as measured by IMAGEMASTER 2D software.

^d^Sequence coverage (%) indicates the number of amino acids spanned by the assigned peptides divided by the sequence length.

^e^Mowse score indicates the probability that the match between the database and a spectrum is a random event.
